The article "Effects of Clopidogrel Rehabilitation on Cardiac Protein Kinase C, Cardiac Heat Shock Protein 70, and CI in MIRI Rat Model" was retracted in 2023. Reasons: suspected computer-generated content; unreliable results or conclusions; concerns about the data; concerns about the results or conclusions.

# Effects of Clopidogrel Rehabilitation on Cardiac Protein Kinase C, Cardiac Heat Shock Protein 70, and CI in MIRI Rat Model

**DOI:** 10.1155/2022/5823276

**Published:** 2022-10-13

**Authors:** Qiaoyan Ma, Lizhong Wang, Hongyan Ma, Qian Cao, Jiagui Ma

**Affiliations:** ^1^Beijing Rehabilitation Hospital of Capital Medical University, Beijing 100144, China; ^2^Dongzhimen Hospital Beijing University of Chinese Medicine, Beijing 101121, China

## Abstract

In order to investigate the effects of clopidogrel rehabilitation on the levels of cardiac protein kinase C (PKC), cardiac heat shock protein 70 (HSP70), and cardiac index (CI) in rats with myocardial ischemia-reperfusion injury (MIRI), sixty Wistar rats are randomly divided into three groups (sham operation group, model group, and clopidogrel group), with 20 rats in each group. The clopidogrel group is given clopidogrel by gavage, and the sham operation group and the model group are given the same amount of normal saline by gavage. The experimental results show that compared with the model group, the clopidogrel group has clear horizontal lines and cell edema. The myocardial infarction rate, creatine kinase-MB (CK-MB), and malondialdehyde (MDA) of the model group and clopidogrel group in the control sham operation group significantly increase.

## 1. Introduction

Myocardial ischemia is a high incidence of clinical cardiovascular disease. Long-term ischemia can cause myocardial cell damage and, in severe cases, myocardial tissue necrosis. Early reperfusion of myocardial blood supply will aggravate myocardial ischemia damage and cause ischemia-reperfusion injury [1]. Development of effective drugs against ischemia/reperfusion injury is a medical problem urgently to be solved in clinical cardiac rehabilitation treatment. In recent years, clopidogrel has been widely used in coronary heart disease and other cardiovascular diseases and has achieved remarkable results. It can effectively improve cardiac function and myocardial injury and has a certain potential research value in ischemia-reperfusion injury [2].

Protein kinase C (PKC) is a calcium-phospholipid-dependent protein kinase involved in cell proliferation, differentiation, and signal transduction. The level of heat shock protein 70 (HSP70) is closely associated with myocardial injury and fibrosis. However, the protective effect of clopidogrel on ischemia-reperfusion injury and the mechanism of HSP70, PKC, and oxidative stress have not been clarified [3]. Therefore, this study constructs a myocardial ischemia-reperfusion injury (MIRI) rat model to further analyze the influence of clopidogrel intervention on MIRI.

The rest of this paper is organized as follows: Section 2 discusses the related works, followed by focusing on the animal model construction and cardiac histopathological examination in Section 3. The myocardial infarction rate and myocardial enzyme indexes are discussed in Section 4.  Section 5 concludes the paper.

The article "Effects of Clopidogrel Rehabilitation on Cardiac Protein Kinase C, Cardiac Heat Shock Protein 70, and CI in MIRI Rat Model" was retracted in 2023. Reasons: suspected computer-generated content; unreliable results or conclusions; concerns about the data; concerns about the results or conclusions.

## 2. Related Works

MIRI was the injury of myocardial cells after the restoration of blood perfusion in ischemic state, which was irreversible, and the body would release a large number of harmful factors such as excitatory amino acids and oxygen free radicals after the occurrence of MIRI [4]. It was speculated that the main mechanism was as follows: malondialdehyde (MDA) was a reaction product of oxygen free radical lipid peroxidation, and superoxide dismutase (SOD) was the main enzyme of oxygen free radical scavenging in the body. Therefore, MDA could be used as a sensitive indicator of oxygen free radical level and lipid peroxidation reaction degree in human body. SOD could reflect the antilipid peroxidation ability of the body to a certain extent, and the levels of both indexes could be used as important reference indexes to evaluate the oxygen free radical content of the body [5]. Clopidogrel was a commonly used platelet receptor blocker in clinical practice. Clopidogrel could inhibit the secretion of inflammatory factors and platelet aggregation, thus exerting obvious anti-inflammatory and antiplatelet effects [6].

HSP70, one of the stress proteins in the body after injury, could be secreted in large quantities, and this index was obviously associated with myocardial ischemia-reperfusion injury [7]. It could inhibit the secretion and expression of HSP70 under the condition of rapid free radical scavenging, which was consistent with the previous studies [8]. HSP70 could be widely used as an indicator to evaluate the occurrence of MIRI and the effect of cardiac rehabilitation. The changes of PKC in the three groups were analyzed, and it was found that the mRNA expression and protein expression of PKC were significantly increased after the occurrence of MIRI and showed a decreasing trend after clopidogrel treatment, indicating that the abnormal increase of PKC was related to the occurrence of MIRI [9].

Clopidogrel could significantly improve atherosclerosis and myocardial infarction and had a good antiplatelet effect [10]. Creatine kinase-MB (CK-MB) was a serum enzyme index for detecting myocardial infarction. CK-MB was mainly distributed in myocardial cells. With the aggravation of myocardial injury, the level of this index increases, which was a better index of myocardial injury. A comprehensive analysis was carried out, and CK-MB of the model group and the clopidogrel group was significantly higher than those of the sham operation group, and the model group was the highest, which verified the above research conclusions, suggesting that the application of clopidogrel could reduce MIRI heart damage and improve heart rate function [11].

The article "Effects of Clopidogrel Rehabilitation on Cardiac Protein Kinase C, Cardiac Heat Shock Protein 70, and CI in MIRI Rat Model" was retracted in 2023. Reasons: suspected computer-generated content; unreliable results or conclusions; concerns about the data; concerns about the results or conclusions.

## 3. Animal Model Construction and Cardiac Histopathological Examination

The rat model of myocardial ischemia/reperfusion is established 2 hours after the last administration. The rats are anesthetized with 25% saccharide (0.4 ml/100 g). Acupuncture needles are inserted subcutaneously into the limbs of the rats, and the normal standard II lead electrocardiogram is recorded. The neck, left chest, and abdomen are all prepared for skin treatment. Endotracheal intubation is performed and connected to the animal ventilator. The frequency is set at 60 times/min, the tidal volume is 15 ml/kg, and the inhalation and inhalation ratio is 1 : 2. Then, the heart is completely exposed and extracted by intercostal thoracotomy along the left sternal margin 3-4, and the left anterior descending coronary artery is ligated with 5/0 needle suture. The obvious elevation of the segment and the dark color of the heart below the ligature line are regarded as the marks of successful coronary artery ligation. Place the heart back in the chest in time and cover the wound with gauze soaked in saline. After 30 min of ischemia, the ligation line is cut off, and the segment decline and the color restoration of the corresponding parts are taken as the start marks of reperfusion. The model is successfully constructed after 60 min of reperfusion. The sham operation group only undergoes suture operation without ligation, and the procedure is the same as the model group and clopidogrel group. The clopidogrel group is given 3 mg/kg clopidogrel by gavage, while the sham operation group and the model group are given the same amount of normal saline by gavage.

After infusion of phosphate buffer, rat heart tissue is taken and fixed with 4% paraformaldehyde. After 24 h, the cells are dehydrated by graded ethanol, and the morphology of the heart tissue is observed under a light microscope.

The heart tissue is extracted and sectioned, placed at 37°C, fixed with formaldehyde after 12 min, and taken by high-definition camera 2 h later and imported into image analysis system to calculate the proportion of infarct area.

The body weight of the rats is weighed. After anesthesia, the heart tissue is extracted and weighed. Cardiac index (CI) (%) is equal to (heart weight/body weight) × 100%.

3 ml blood samples are centrifuged for 15 min at the speed of 12 000 r/min, and the supernatant is collected by centrifuge tube and stored in freezer for inspection. The CK-MB and troponin (Tn) levels are determined by using an automatic biochemical analyzer, and the method is Lai-colorimetric method.

The article "Effects of Clopidogrel Rehabilitation on Cardiac Protein Kinase C, Cardiac Heat Shock Protein 70, and CI in MIRI Rat Model" was retracted in 2023. Reasons: suspected computer-generated content; unreliable results or conclusions; concerns about the data; concerns about the results or conclusions.

SOD and MDA are determined by fluorescence detection method, and the kits are purchased from Biyuntian Reagent Company. The reagents and standard substances are mixed strictly according to the instructions and then placed in water bath at 95°C for 40 min. The serum is centrifuged at 3 500 r/min for 10 min, and the absorbance is determined.

The myocardial tissues of rats in each group are ground with an appropriate amount of liquid nitrogen, and total ribonucleic acid (RNA) is extracted according to the instructions of mirVana microRNA Isolation Kit, and RNA concentration and purity are detected. Deoxyribonucleic acid (DNA) is obtained by reverse transcription reaction, and quantitative real-time PCR (QR-PCR) reaction system is used to extract DNA and configure HSP70 and PKC. With *β*-actin as internal reference, the target gene sequence and PCR primer synthesis are completed by the laboratory.

Sample tissue is thoroughly ground and 200 *μ*l cracking buffer is added, ice bath is performed for 30 min, and centrifugation is performed at 4°C and 1300 r/min speed for 10 min. The supernatant is extracted and the protein concentration is detected.

Sixty clean Wistar rats are purchased from Beijing Huafukang Biological Company as the research object and are divided into sham operation group, model group, and clopidogrel group according to random number table method, with 20 rats in each group. All rats are female and weighed 275~330 g. The average body weight of sham group, model group, and clopidogrel group is 320.12 ± 3.23 g, 319.12 ± 3.21 g, and 321.12 ± 3.20 g, and there is no statistical difference in body weight between groups (*P* > 0.05).

SPSS 26.0 software is used for statistical analysis. The mean ± standard deviation ($\overset{¯}{x}\pm s$) is used to represent the measurement data of normal distribution. The *t* test is used, and the data between multiple groups is tested using *F* test.

## 4. Myocardial Infarction Rate and Myocardial Enzyme Indexes

### 4.1. Pathological Morphology of Cardiac Tissue

Figure 1 is the pathological morphology of cardiac tissue. It is clearly evident from Figure 1 that in the sham operation group, the cells are orderly arranged with complete structure and clear transverse lines. In the model group, the cells are necrotic and disordered, and in the clopidogrel group, the transverse lines are clearer and there is cell edema.

### 4.2. Myocardial Infarction Rate and Cardiac Index

Table 1 is the pathological morphology of cardiac tissue. It is clearly evident from Table 1 that the myocardial infarction rate of the model group and clopidogrel group is significantly higher than that of the sham group, and the model group is the highest.

The article "Effects of Clopidogrel Rehabilitation on Cardiac Protein Kinase C, Cardiac Heat Shock Protein 70, and CI in MIRI Rat Model" was retracted in 2023. Reasons: suspected computer-generated content; unreliable results or conclusions; concerns about the data; concerns about the results or conclusions.

Figure 2 is the myocardial infarction size and cardiac index. It is clearly evident from Figure 2 that the CI of the model group and clopidogrel group is significantly lower than that of the sham group, and the model group is the lowest, with statistical differences (*P* < 0.05).

### 4.3. Myocardial Enzyme Indexes

Table 2 is the myocardial enzyme indices. It is clearly evident from Table 2 that cTn and CK-MB in the model group and clopidogrel group are significantly higher than those in the sham group.

Figure 3 is the myocardial enzyme indices. It is clearly evident from Figure 3 that cTn and CK-MB are the highest in the model group, with statistical differences (*P* < 0.05).

### 4.4. Oxygen Radical Index

Table 3 is the oxygen radical index. It is clearly evident from Table 3 that MDA in model group and clopidogrel group is significantly higher than that in sham group.

Figure 4 is the oxygen radical index. It is clearly evident from Figure 4 that SOD in model group and clopidogrel group is significantly lower than that in sham group and the lowest in model group, with statistical differences (*P* < 0.05).

Table 4 is the HSP70 and PKC mRNA expression levels. It is clearly evident from Table 4 that the mRNA levels of HSP70 and PKC in model group and clopidogrel group are significantly higher than those in sham group and the highest in model group, with statistical differences (*P* < 0.05) (see Table 4 and Figure 5).

Figure 5 is the HSP70 and PKC mRNA expression levels. It is clearly evident from Figure 5 that the mRNA levels of HSP70 and PKC in model group are the highest, with statistical differences (*P* < 0.05).

Table 5 is the protein expression of HSP70 and PKC. It is clearly evident from Table 5 that the protein levels of HSP70 and PKC in model group and clopidogrel group are significantly higher than those in sham operation group.

Figure 6 is the protein expression of HSP70 and PKC. It is clearly evident from Figure 6 that the protein levels of HSP70 and PKC in model group are the highest, with statistical differences (*P* < 0.05).

## 5. Conclusion

HSP70 and PKC are abnormally elevated in MIRI, and clopidogrel treatment can improve the cardiac function and myocardial infarction of MIRI, quickly remove free radicals, and inhibit the expression of HSP70 and PKC, thus reducing the myocardial injury caused by HSP70 and PKC. The experimental results show that compared with the sham operation group, the MIRI model rats have significantly lower SOD and significantly higher MDA levels, and the clopidogrel group is better than the model group, further indicating that the occurrence of MIRI can stimulate the body to overproduce oxygen free radicals, while clopidogrel can effectively scavenge oxygen free radicals.

The article "Effects of Clopidogrel Rehabilitation on Cardiac Protein Kinase C, Cardiac Heat Shock Protein 70, and CI in MIRI Rat Model" was retracted in 2023. Reasons: suspected computer-generated content; unreliable results or conclusions; concerns about the data; concerns about the results or conclusions.

## Figures and Tables

**Figure 1:** Pathological morphology of cardiac tissue: (a) operation group; (b) model group; (c) clopidogrel group.

**Figure 2:** Myocardial infarction size and cardiac index.

**Figure 3:** Myocardial enzyme indices.

**Figure 4:** Oxygen radical index.

**Figure 5:** HSP70 and PKC mRNA expression levels.

**Figure 6:** Protein expression of HSP70 and PKC.

**Table 1:** Myocardial infarction size and cardiac index ($\overset{¯}{x}\pm s$, *n* = 20).

Group	Cardiac infarction rate (%)	CI (min·m^2^)
Sham group (*n* = 20)	0.56 ± 0.14	3.56 ± 0.54
Model group (*n* = 20)	22.21 ± 7.43^∗^	2.51 ± 0.43^∗^
Clopidogrel group (*n* = 20)	15.33 ± 4.22^∗^^#^	3.03 ± 0.34^∗^^#^
*F*	12.211	4.343
*P*	0.000	0.000

**Table 2:** Myocardial enzyme indices ($\overset{¯}{x}\pm s$, *n* = 20).

Group	cTn (*μ*g/l)	CK-MB (U/l)
Sham group (*n* = 20)	21.56 ± 5.14	47.76 ± 7.54
Model group (*n* = 20)	35.51 ± 7.43^∗^	229.32 ± 24.21^∗^
Clopidogrel group (*n* = 20)	27.33 ± 6.34^∗^^#^	25.56 ± 5.45^∗^^#^
*F*	8.565	9.766
*P*	0.000	0.000

**Table 3:** Oxygen radical index ($\overset{¯}{x}\pm s$, *n* = 20).

Group	SOD (U/ml)	MDA (nmol/ml)
Sham group (*n* = 20)	343.56 ± 35.14	147.76 ± 17.54
Model group (*n* = 20)	135.51 ± 23.43^∗^	329.32 ± 20.21^∗^
Clopidogrel group (*n* = 20)	227.33 ± 26.34^∗^^#^	225.56 ± 25.45^∗^^#^
*F*	13.221	10.232
*P*	0.000	0.000

**Table 4:** HSP70 and PKC mRNA expression levels ($\overset{¯}{x}\pm s$, *n* = 20).

Group	HSP70 mRNA	PKC mRNA
Sham group (*n* = 20)	1.02 ± 0.04	1.06 ± 0.09
Model group (*n* = 20)	1.51 ± 0.06^∗^	1.42 ± 0.21^∗^
Clopidogrel group (*n* = 20)	1.33 ± 0.34^∗^^#^	1.21 ± 0.15^∗^^#^
*F*	15.343	12.553
*P*	0.000	0.000

**Table 5:** Protein expression of HSP70 and PKC ($\overset{¯}{x}\pm s$, *n* = 20).

Group	HSP70 protein	PKC protein
Sham group (*n* = 20)	0.82 ± 0.14	0.92 ± 0.09
Model group (*n* = 20)	1.72 ± 0.09^∗^	1.32 ± 0.15^∗^
Clopidogrel group (*n* = 20)	0.93 ± 0.10^∗^^#^	1.13 ± 0.11^∗^^#^
*F*	11.433	10.232
*P*	0.000	0.000

## Data Availability

The simulation experiment data used to support the findings of this study are available from the corresponding author upon request.
